# A Study on the Association between Korotkoff Sound Signaling and Chronic Heart Failure (CHF) Based on Computer-Assisted Diagnoses

**DOI:** 10.1155/2022/3226655

**Published:** 2022-09-01

**Authors:** Huanyu Zhang, Ruwei Wang, Hong Zhou, Shudong Xia, Sixiang Jia, Yiteng Wu

**Affiliations:** ^1^College of Biomedical Engineering & Instrument Science, Zhejiang University, Hangzhou 310013, China; ^2^The Fourth Affiliated Hospital Zhejiang University School of Medicine, Zhejiang University, Yiwu 322000, China

## Abstract

**Background:**

Korotkoff sound (KS) is an important indicator of hypertension when monitoring blood pressure. However, its utility in noninvasive diagnosis of Chronic heart failure (CHF) has rarely been studied.

**Purpose:**

In this study, we proposed a method for signal denoising, segmentation, and feature extraction for KS, and a Bayesian optimization-based support vector machine algorithm for KS classification.

**Methods:**

The acquired KS signal was resampled and denoised to extract 19 energy features, 12 statistical features, 2 entropy features, and 13 Mel Frequency Cepstrum Coefficient (MFCCs) features. A controlled trial based on the VALSAVA maneuver was carried out to investigate the relationship between cardiac function and KS. To classify these feature sets, the K-Nearest Neighbors (KNN), decision tree (DT), Naive Bayes (NB), ensemble (EM) classifiers, and the proposed BO-SVM were employed and evaluated using the accuracy (Acc), sensitivity (Se), specificity (Sp), Precision (Ps), and F1 score (F1).

**Results:**

The ALSAVA maneuver indicated that the KS signal could play an important role in the diagnosis of CHF. Through comparative experiments, it was shown that the best performance of the classifier was obtained by BO-SVM, with Acc (85.0%), Se (85.3%), and Sp (84.6%).

**Conclusions:**

In this study, a method for noise reduction, segmentation, and classification of KS was established. In the measured data set, our method performed well in terms of classification accuracy, sensitivity, and specificity. In light of this, we believed that the methods described in this paper can be applied to the early, noninvasive detection of heart disease as well as a supplementary monitoring technique for the prognosis of patients with CHF.

## 1. Introduction

Blood pressure monitoring that makes use of Korotkoff sound (KS) has been widely utilized to detect potential hypertension in patients [1–3]. KS enables shorter test duration, simple processing, and strong anti-interference capabilities and has clear signal characteristics. Because of these advantages, meticulous experimental methods and diagnostic algorithms will enable the early nondestructive diagnosis of cardiovascular disease [4, 5]. The characteristics of KS can be divided into a short, rapid impact, followed by a rumble or murmur. Lange and Hecht [6] found that KS was accompanied by a sharp drop in cuff pressure. They believed that KS was caused by brachial artery vibration. Toward this end, Rodbard and Robbins [7] used an experimental model to simulate KS. This set of experiments supported a connection between a sudden drop in cuff pressure and the opening of the brachial artery. Researchers have since found that blood flow also plays an important role in the development of KS. Sykes et al. [8] used real-time two-dimensional ultrasound and Doppler techniques to study Bradley artery movements and blood flow turbulence during blood pressure measurement. Here, the KS was hypothesized to be derived from large oscillations in the brachial artery and flow turbulence in the blood. Benmira et al. [9] performed a detailed analysis of KS and ECG signals using B-mode and duplex ultrasonography and concluded that KS resulted from the pounding produced by the vibration of an arterial wall and the rumbling produced by the turbulence of blood flow.

Accordingly, the KS mechanism might be directly or indirectly related to the state of the arteries and the state of the heart. Gosse et al. [10] used the time interval of KS (QKD) and parameters of the equivalent KS interval (QKD_h_) to study associations between KS and arteriosclerosis, heart disease, and stroke. The authors found a strong association between QKD_h_ and cardiovascular disease, which is suggested to be used as a diagnostic basis for stroke. Ormerod et al. [11] found that QKD parameters were strongly associated with stroke caused by aortic sclerosis, while the relationships between cardiac embolism and small artery occlusion subtypes were not clear. Ramakrishnan [12] studied the effects of age and gender on the amplitude of KS, suggesting that the amplitude of KS could be used to predict atherosclerosis. These studies have shown that KS indirect features could be used to prove that there is a strong association between arteriosclerosis and cardiovascular disease. However, studies on the direct association between KS′ direct features, such as time-frequency characteristics, and heart disease have rarely been carried out.

It is vital to note that one of the most significant noncommunicable diseases that endanger human life and health is heart disease [13], particularly CHF. Heart disease patients have grown dramatically in number during the past few decades, particularly in economically poor regions. However, the diagnosis of CHF is a time-consuming process that necessitates expensive medical equipment, making it an unaffordable burden for the majority of low-income people. This considerably increases the risk of the condition, making it more difficult to treat and prevent chronic heart failure. With the development of machine learning (ML) technology in the medical field [14, 15], an effective, cheap solution for the prediagnosis of CHF has been possible.

The identification and categorization of heart sound (HS) have received the majority of research attention in the area of cardiac disease prediagnosis. [16] The noise reduction, preprocessing, and classification of enormous volumes of HS data using machine learning algorithms have produced outstanding results in these studies. [17, 18] However, the professionalism of the HS acquisition procedure severely limits the adoption of this technology in the general population.

The objective of this project is to increase the probability of early detection of CHF disease through the study of prediagnosis of CHF, to improve the quality of life of potentially high-risk people with CHF. In consideration of the widespread use of the KS method in blood pressure monitoring, this paper proposed a time-frequency analysis technology and machine learning algorithm to investigate Chronic heart failure (CHF) classification based on KS time-frequency features. This method will be used to establish a clear relationship between KS and CHF. The method described in this paper is divided into four steps:

1. Noise reduction of KS signals using the Wiener filtering method
2. Energy envelope-based signal segmentation
3. Signal feature extraction based on time-frequency analysis method
4. KS Signal classification utilizing ML algorithms.

This article aims to establish a practical and noninvasive prediagnosis method that is highly conducive to promotion among individuals without medical expertise. The primary contributions of this work can be summarized as follows:

- A KS-specific denoising, segmentation, and feature extraction approach was created.
- The Valsalva maneuver was used to demonstrate the association between KS signal features and CHF, and the direct correlation between KS signals and CHF was established.
- The energy features, statistical features, entropy features, and MFCCs features of KS signals were extracted, and the effects of different features on classification performance were investigated by the ML algorithm.
- The feasibility of the KS signals in early CHF diagnosis was demonstrated using a feature extraction technique and a machine learning algorithm, providing a novel technical route for convenient and noninvasive CHF diagnosis.

## 2. Related Works

Due to the shortage of studies on the automatic classification of KS signals, we will use HS detection methods for cardiac disorders as the inquiry object to examine the current research progress. HS-based diagnosis of cardiac diseases involves signal noise reduction, signal segmentation, feature extraction, and classification. [18].

Noise reduction has become an important aspect of HS signal processing due to environmental noise, electromagnetic noise, power frequency noise, human breath sound, lung sound, and other factors. Reasonable noise reduction will improve the signal-to-noise ratio of audio and the diagnostic model's accuracy. Wavelet denoising, empirical mode decomposition denoising, adaptive denoising, singular value decomposition (SVD) denoising, and combination approaches are all commonly used noise reduction methods. [19] Mondal et al. [20] introduced an HS denoising method based on a combined framework of wavelet packet transform (WPT) and SVD. The experimental study showed that their method was more reliable and robust than the industry standard method. Deng and Han [21] proposed an adaptive denoising algorithm, which did not need the predefined base function and can be performed in an adaptive way for different noise levels and group sizes. Compared with the conventional wavelet methods, this algorithm had a better denoising effect at low noise levels.

HS signal segmentation is a commonly used method for HS signal feature extraction, such as envelope-based methods, feature-based methods, machine learning approaches, and hidden Markov model (HMM) based methods. The accuracy of the classification model will be significantly influenced by signal segmentation technology, so researchers had invested many efforts to increase the accuracy of signal segmentation. Thalmayer et al. [22] proposed an envelope-based approach that was evaluated using two distinct methods for extracting envelope curves: the Hilbert transform and the short-time Fourier transform. The classification results revealed that the Hilbert transform performed better in terms of F1 score and computing effort, achieving an F1 score of up to 95.7% and an average of 90.5% for the S1 classification. Giordano and Knaflitz [23] employed the Shannon energy envelope algorithm to perform a reliable quantitative characterization of the timing of the occurrence of HS components; they believed that this method was more efficient than other energy envelope methods due to the lack of a search-back phase in the HS detection process. Springer et al. [24] proposed an enhanced hidden Markov algorithm for HS signal segmentation, which included duration dependencies and logistic regression-based emission probabilities, and the implementation of an extension to the Viterbi algorithm for use with hidden semi-Markov models (HSMMs). Li et al. [25] used the Empirical Wavelet Transform (EWT) to decompose S1 and the Hilbert Transform to extract the instantaneous frequency (IF) of the mitral component (M1) and the tricuspid component (T1). Chen et al. [26] proposed a deep neural network (DNN) method for recognizing S1 and S2 HS by MFCCs.

The development of machine learning algorithms promotes the advancement of heart disease prediagnosis technology. A large number of algorithms and models have been presented for the diagnosis of cardiac disease. [27] Potes et al. [28] identified heart sounds with an integrated algorithm and a deep learning algorithm, reaching 86% classification accuracy on the 2016 PhysioNet/CinC Challenge database. Since then, an increasing number of researchers have focused on the identification of cardiac disease using heart sounds. Juniati et al. [29] used the Higuchi Algorithm to calculate the fractal dimension of the HS and classified fractal dimension by KNN and Fuzzy c-mean clustering methods, and the best accuracy obtained was 86.17% based on the proposed method. Noman et al. [30] proposed a Markov-switching autoregressive with a switching linear dynamic system (MSAR-SLDS) to model the raw HS signals and extracted 37 MFCCs features and 16 time and frequency-domain features; finally, using HMM on the large 2016 PhysioNet/CinC Challenge database, a classification accuracy of 86.1% was obtained. Nogueira et al. [31] proposed a methodological combination of time domain and frequency domain features of phonocardiogram signals to improve cardiac disease automatic classification. Using an SVM radial basis algorithm, they obtained an accuracy of approximately 83.22%. Shi et al. [32] collected the HS signal through radar technology and extracted the Springer Features and Custom Features. For classification research, the proposed Ensemble (EM) Classifiers were used, and they achieved a classification accuracy of 96.36%.

Gjoreski et al. [33] established a CHF detection approach based on heart sounds using filtering, segmentation, feature extraction, and machine learning. Their method, which was based on data from 122 subjects, had a 96% classification accuracy and an 87% detection accuracy for CHF. A few years later, Gjoreski et al. [34] used a combination of classical machine learning and an end-to-end deep learning model to classify 947 subjects in six public HS datasets and one collected CHF dataset, achieving a 92.9 % classification accuracy. Zheng et al. [35] extracted time-domain, frequency-domain, and nonlinear features to build multiscale and multidomain heart sound features and achieved a classification accuracy of 82% using a least-squares support vector machine (LS-SVM).

Prediagnosis of heart disease has also yielded impressive results in the field of non-heart sound monitoring. Reddy et al. [36] used an adaptive genetic algorithm with fuzzy logic (AGAFL) model to predict heart disease, and the experimental results showed that the classification accuracy of this method was obviously better than that of the existing Rule Based Fuzzy Logic Classifier with Locality Preserving Projection (LPP-RBFL) and Fuzzy Logic Classifier with Rough Set algorithm (RS-FL). Hussain et al. [37] used support vector machine (SVM), decision tree (DT), K-nearest neighbors (KNN), and ensemble (EM) classifiers for CHF detection by collecting multimodal features to capture temporal, spectral, and complex dynamics features, with the SVM linear kernel providing the best classification accuracy of 93.1%. Ali et al. [38] proposed the hybrid grid search algorithm (HGSA) to optimize an SVM model for CHF detection, achieving 92.22% accuracy. A few years later, Ali and Bukhari [39] proposed a two-stage decision support system based on mutual information (MI) and the optimal neural network configuration to overcome overfitting and optimize the generalization factor. According to their suggested method, the best accuracy was up to 93.3%.

## 3. Methods and Materials

### 3.1. System Overview

Figure 1 gives an overview of the proposed system's functionality. Firstly, the collected signals are preprocessed, which includes resampling, noise reduction, and signal recognition. Then, the features of the sound signal are analyzed, in order to extract the effective features. This involves sound signal segmentation, wavelet packet (WP) decomposition, feature extraction, and feature regularization.

Given that the KS signal consists of a group of rapid and short-pulse sound, the accurate extraction of feature sets is the focus of the current study. In addition, there are significant differences in the signal length between different groups of people, so the characteristic data set needs to be normalized using a root mean square value, maximum value, and minimum value. Finally, the signal feature sets are fed into the ML models for training and prediction, to ultimately diagnose CHF.

### 3.2. Participants

A total of 300 subjects were selected. As shown in Table 1, the study included 115 healthy subjects aged 22 to 63 years old, with systolic blood pressures ranging from 96 to 126 mm Hg and diastolic blood pressures ranging from 63 to 84 mm Hg. CHF patients ranged in age from 43 to 79 years old, with systolic blood pressure ranging from 94 to 164 mm Hg and diastolic blood pressure ranging from 57 to 98 mm Hg. Those with CHF had a left ventricular ejection fraction that was less than 50%, and all selected patients were evaluated by experienced cardiologists.

Before the KS signal acquisition process, subjects were fully aware of the testing procedures and asked to sign authorization forms. All subjects were anonymous. The data collection process was completed using standard testing equipment within the Department of Cardiology at the Fourth People's Hospital of Zhejiang University. The study was authorized by the Ethics Committee of Zhejiang University.

### 3.3. Data Processing Process

We carried out preprocessing of data through signal denoising, signal location, signal segmentation, feature extraction, etc. A flowchart of KS is shown in Figure 2.

### 3.4. Wiener Filtering

Wiener filtration is a denoising method based on the minimum error between the predicted result and the true value. The basic working principle of Wiener filtration is as follows (Figure 3) [40]:where *s*(*n*) is a pure sound signal, and *d*(*n*) is a noise signal. The Wiener filtration algorithm requires a digital filter. Assuming the input signal is *y*(*n*), the output of the filter is as follows:

(1) $$\begin{array}{c} s^{\prime }\left(n\right)=y\left(n\right)\cdot h_{n}=\sum_{m=-\infty }^{+\infty }y\left(n-m\right)\cdot h_{m}, \end{array}$$

where *h*_*m*_ is the filter coefficient vector.

The least root mean square error criterion, as given in the formula (2), is used in Wiener filtering to ensure that the output signal is as similar to the original signal as possible.

(2) $$\begin{array}{c} E\left\{e^{2}\right\}=E\left\{{\left(s-x\cdot h\right)}^{2}\right\}=\min. \end{array}$$

### 3.5. Shannon Envelope

Due to its excellent processing efficiency and noise-resistance, the Shannon energy method has emerged as one of the most commonly used segmentation algorithms for HS [23]. Based on these advantages, we decided to use the Shannon energy envelope algorithm for KS segmentation in this paper. The KS signal was truncated into multisegment, 40 ms signal set for the calculation, and the signal's envelope was calculated using a window with a 50% overlap. The Shannon energy of each segment is defined as follows [41]:

(3) $$\begin{array}{c} E_{j}=-\frac{1}{N}\sum_{i=1}^{N}Z_{i}{}^{2}\cdot \;\log\;Z_{i}{}^{2}, \end{array}$$

where *Z*_*i*_ is normalized intercepted signal, *Z*_*i*_ = *x*_*i*_/max|*x*_*i*_|. *x*_*i*_ is the intercepted signal.

Then, Shannon energy was normalized *via* (4) to obtain the normalized Shannon energy.

(4) $$\begin{array}{c} Pj=\frac{E_{j}-\text{mean}\left(E_{j}\right)}{\text{std}\left(E_{j}\right)}. \end{array}$$

According to some studies, normalized average Shannon energy is sensitive to noise, which can lead to false segmentation. Signal segmentation is more difficult with KS, because valuable signals and high-intensity murmurs always overlap. Although the high-order Shannon technique can further minimize murmurs, it can also prevent valuable signals from being identified [42], particularly in the early stages of KS. Fortunately, the Wiener filtering method we used successfully minimizes the noise level and overcomes the problem with the Shannon energy approach in KS signal segmentation. The extraction effect diagram of the Shannon energy envelope for the KS is shown in Figure 4(b).

### 3.6. Location and Segmentation

A peak signal was taken as a benchmark for locating the sound, and a threshold value was set at 0.2x the maximum peak within the envelope of the sound signal. Overlocalization occurred when multiple peaks in a single KS signal caused localization error, which compounded subsequent calculation inaccuracies. In addition, due to the interference of factors such as the friction between the stethoscope diaphragm and the skin, arm swing, and other factors, abnormal wide-band noise often occurred at the beginning and end of the KS signal. These interfering elements can greatly occlude the signal recognition process. Thus, it is necessary to recheck results at each step to eliminate invalid information such as abnormal anchor points and overlocalization anchor points. The following criteria were designed for signal recognition:

1. If the time interval between two anchor points was less than 100 ms, these anchor points would be combined into a single anchor point;
2. There will be a period of silence before the KS appears and after it disappears during the KS test. The silent phase should be noiseless. However, due to the friction between the skin and the microphone, the signals we collected frequently contained aberrant pulse noises, which should be recognized and eliminated by signal segmentation.

Here, the starting point of the KS signal began with the anchor point and searched forward for 300 ms. The ending point of the KS signal began with the anchor point and searched backward for 500 ms. The segmentation results of the identified energy envelopes within the KS signal are shown in Figures 4(c) and 4(d), where B means the beginning of the KS, and E means the ending of the KS.

### 3.7. Feature Extraction

We extracted a total of 47 features for each KS signal, including 19 energy features, 12 statistics features, 2 entropy features, and 13 MFCCs features. The feature extraction procedure was as follows:

#### 3.7.1. Energy-Based Features

Based on WP coefficients, the energy distribution of each signal component was extracted. The statistical energy formula based on the WP analysis is as follows: [43].

(5) $$\begin{array}{c} E\left(i,j\right)=\int {\left|S_{i,j}\right|}^{2}\text{d}t=\sum_{k=0}^{2^{j}-1}{\left|x_{j,k}\right|}^{2}, \end{array}$$

where *E*(*i*,*j*) is the energy of the WP, and *x*_*j*,*k*_ is the wavelet coefficient.

Unlike HS or other stable signals, the duration of the KS signal varies from person to person, resulting in a large variation in the length of the test data. A three-layer WP decomposition was carried out on all effective KS signals. As a result, 8 groups of wavelet coefficients were obtained, and the ratio of energy of each wavelet coefficient to total energy was calculated, using formula (6). This set of data was defined as the global energy ratio, or *S*_total_(50–100), *S*_total_(100–150), *S*_total_(150–200), *S*_total_(200–250), *S*_total_(250–300), *S*_total_(300–350), and *S*_total_(350–400).

(6) $$\begin{array}{c} S\_\text{total}\left(j\right)=\frac{E\left(j\right)}{E_{\text{total}}}, \end{array}$$

where *E*(*j*) is the energy of each wavelet coefficient, and *E*_total_ is sum of the energies of all the wavelet coefficients.

Each individual KS signal was decomposed by the WP, and each WP coefficient energy ratio was calculated by (7) and (8). Here, the energy ratio within 50–100 Hz is defined as the ratio of low frequency energy (*e*_*n*_); the energy ratio within 100–400 Hz is defined as high frequency energy (*e*_*n*_*h*_); and the energy ratio within 50–400 Hz is defined as total energy (*E*_*t*_).

(7) $$\begin{array}{c} e_{n}=\frac{E_{n\left(50-100\text{ Hz}\right)}}{E_{n\text{ total}\left(50-400\text{ Hz}\right)}}, \end{array}$$

(8) $$\begin{array}{c} e_{n\_h}=\frac{E_{n\left(150-400\text{ Hz}\right)}}{E_{n\text{ total}\left(50-400\text{ Hz}\right)}}. \end{array}$$

Here, *E*_*n*(50 − 100 Hz)_ is the energy within 50–100 Hz of each individual KS signal; *E*_*n*(150 − 400 Hz)_ is the energy within 150–400 Hz of each individual KS signal; and *E*_*n* total(50 − 400 Hz)_ represents the total energy of each individual KS signal.

The variability of the KS energy ratio and time interval was calculated using (9)–(12), in order to study the influence of CHF on KS energy and the time interval.

(9) $$\begin{array}{c} e_{nr}=\frac{e_{n}}{\sum_{i=1}^{n}e_{n}}n, \end{array}$$

(10) $$\begin{array}{c} e_{nr\_h}=\frac{e_{n\_h}}{\sum_{i=1}^{n}e_{n\_h}}n, \end{array}$$

(11) $$\begin{array}{c} E_{p}=\frac{E_{t}}{\sum_{i=1}^{n}E_{t}}n, \end{array}$$

(12) $$\begin{array}{c} TM=\frac{Ti}{\sum_{i=1}^{n}Ti}n, \end{array}$$

where *n* is the number of all KS signals in a data set, and *Ti* is time interval between each KS signal. A total of 19 energy-based features are obtained after extracting each KS signal according to the description given above.

#### 3.7.2. Statistical Features

Statistical parameters of each KS signal were extracted: mean, median, standard deviation, mean absolute deviation, 1st quartile, 3rd quartile, interquartile range, skewness, kurtosis, dominant frequency, dominant frequency magnitude, and dominant frequency ratio.

#### 3.7.3. Entropy Features

Signal entropy, as a nonlinear property, reflects the complexity of a set of time series signals. The signal's entropy increases with its effective information content. In this study, the signal entropy and frequency entropy of a KS signal were extracted, and the signal entropy and frequency entropy were stated as follows [44]:

(13) $$\begin{array}{c} H_{s}=-\sum p\left(x\right)\log\left(p\left(x\right)\right). \end{array}$$

When computing the signal entropy, *p*(*x*) is the probability that the signal *x* falls in the time domain *X*(*L*), and *X* (*L*) represents the KS time domain interval. When computing frequency entropy, *p*(*x*) is the probability that the signal *x* falls in the frequency domain *Z*(*L*), and *Z* (*L*) is the KS frequency domain interval.

#### 3.7.4. Mel Frequency Cepstrum Coefficient

Mel frequency is a speech spectra simulating human hearing. The energy signal output is created by constructing several groups of Mel filters, which are independent of the original signal. The MFCCs algorithm is more suitable for the auditory characteristics of human hearing, and it still performs well when the signal-to-noise ratio is low. The decorrelated Mel cepstrum coefficients are expressed as follows using the discrete cosine transform (DCT) [45]:

(14) $$\begin{array}{c} MFCCs\left(n_{1}\right)=\sum_{m=1}^{M}\log\left[E\left(m,k\right)\right]\cdot \;\cos\left(\frac{\left(m-0.5\right)}{M}\cdot n_{1}\cdot \pi \right),\;n_{1}=1,2,\ldots ,L, \end{array}$$

where *n*_1_ is the order of MFCCs, M is the number of triangular filters, and *E*(*m*, *k*) is the output energy generated by the Mel filter. From each KS signal, we extract 13 Mel cepstrum features.

### 3.8. Support Vector Machine (SVM) Based on Particle Swarm Optimization

SVM is an efficient machine learning method based on statistical learning theory, which was first proposed by Cortes and Vapnik [46, 47]. The main objective is to establish a classified hyperplane as the decision surface, in order to maximize the distance between positive and negative examples [37]. In SVMs, a kernel function *g* and penalty function *c* have great influence on the selection of a hyperplane; they are also the key to determining the classification accuracy. At present, there is no recognized optimal method to select the appropriate kernel function and penalty function, so this study has been designed, in part, to solve this problem by using a Bayesian optimization algorithm.

The Bayesian optimization (BO) algorithm is an efficient optimization algorithm because it utilizes prior beliefs to help direct the sampling of the object and to trade off exploration and exploitation of the search space [48, 49]. The BO algorithm utilizes the Bayesian theorem to find the parameters that make the objective function globally optimal through known prior information. According to the theory, for a given event *E*, the posterior probability *P*(*M*|*E*) of model *M* is proportional to the likelihood probability to *P*(*E*|*M*) of *E* given *M* multiplied by the a priori probability *P*(*M*) of *M* [49], as shown as follows:

(15) $$\begin{array}{c} P\left(M|E\right)\propto P\left(E|M\right)P\left(M\right). \end{array}$$

Many studies have shown that the BO algorithm is suitable for expensive and time-consuming optimization tasks; when combined with the SVM algorithm, it will significantly enhance the computational efficiency, classification accuracy, and generalization ability of the SVM model. [50, 51].

### 3.9. K-Nearest Neighbors Classification Algorithm

The KNN algorithm is one of the most widely used in machine learning. Its basic classification principle is to use given samples as a reference, calculate the distance between unknown samples and given samples, and then choose the K closest given samples to the unknown samples. The unidentified samples and the Nearest neighbor samples are put into the same group using the majority-vote voting criterion. The major principles of the KNN algorithm are as follows [29]: to begin, select the K value, which should be an odd integer to ensure the classification's accuracy. Second, determine the distance between two samples; the distance function chosen has a significant impact on the KNN classification performance. Finally, classification rules: the majority-voting voting rule is the most commonly used classification rule in the KNN.

### 3.10. Naive Bayes Classification Algorithm

The Naive Bayes (NB) classification is a classification method based on the Bayesian theorem and independent assumption of feature conditions. The algorithm is simplified based on the Bayesian algorithm, which assumes that when the target value is given, the attributes are conditionally independent of each other. Based on the known prior probability, the primary procedure of this method is to estimate the posterior probability of variables belonging to a specific category. For the given training data, Naive Bayes first learns the joint probability distribution of input and output based on the independent assumption of feature conditions and then applies the Bayesian theorem to determine the maximum posterior probability based on this distribution for new examples.

### 3.11. Decision Tree Classification Algorithm

The DT algorithm is a method of approximating discrete function values by classifying data using a set of criteria. The DT has the advantages of visual interpretability and statistical rigor, which promote the improved design of classification algorithm models [52]. DT creation method can be divided into two steps: the decision tree is first generated by the training sample set. Then, the decision tree generated in the previous stage is tested, corrected, and trimmed. Test data is used to validate the decision tree's production rules, and the branches that affect prebalance accuracy are pruned to improve the decision tree's accuracy and model performance.

### 3.12. Ensemble Learning Classification Algorithm

EM learning is an algorithm for solving learning tasks by constructing several machine learners, which can be used for classification problems, regression problems, feature selection, outlier identification, etc. [53]. For training set data, we can create an enhanced learner by training several independent learners and designing a classifier combination strategy. Two issues must be considered while utilizing EM learning: first, how to gather a large number of individual learners; second, how to select a combination strategy to integrate these individual learners into a powerful learner. Individual learners usually have two options: one is that all individual learners are of the same type, known as homogeneous individual learners, and the other is that all individual learners are not exactly of the same type, known as heterogeneous individual learners. Additionally, EM learning can be classified into bagging algorithm, boosting algorithm, stacking algorithm, etc. based on various combination strategies.

### 3.13. Evaluation Metrics

For the binary classification task, we will obtain four classification results. When a positive sample is correctly classified, we call it a true positive signal (TP), while an incorrectly classified-positive sample is called a false negative signal (FN). When a negative sample is correctly identified, we call it a true negative signal (TN). On the other hand, it is defined as a false positive signal (FP) [54]. Accuracy (Acc), sensitivity (Se), specificity (Sp), Precision (Ps), and F1 score (F1) were introduced as evaluation metrics for classifying KS in order to evaluate each classifier's performance [55], defined as follows:

(16) $$\begin{array}{c} \text{Acc}=\frac{\text{TP}+\text{TN}}{\text{TP}+\text{FN}+\text{TN}+\text{FP}},\\ \text{Se}=\frac{\text{TP}}{\text{TP}+\text{FN}},\\ \text{Sp}=\frac{\text{TN}}{\text{TN}+\text{FP}},\\ \text{Ps}=\frac{\text{TP}}{\text{TP}+\text{FP}},\\ \text{F}1=2\cdot \frac{\text{Se}\cdot \text{Ps}}{\text{Se}+\text{Ps}}. \end{array}$$

## 4. Result

### 4.1. Sensitivity Study

It is widely hypothesized that KS is a result of interactions between blood flow and the brachial artery. The current study investigates how changes in cardiac output may impact brachial artery KS.

The Valsalva maneuver [56], which is commonly used in clinics, has been utilized to simulate abnormal states of cardiac function and reduce the cardiac ejection volume artificially. Specifically, the Valsalva maneuver involves a deep inhalation followed by a forced exhalation while still in the holding state. Doing so can effectively increase pressure in the chest, reduce venous return, and change the volume of blood transfusion to the heart. In this study, ejection volume to the heart was modified in the same volunteer. The hypothesis was that this intervention would effectively eliminate interference factors such as sex, age, and health status and enable control of cardiac ejection volume as a single variable.

Figure 5 shows a comparison of KS time frequency diagrams before and after Valsalva-related action. It can be seen that the KS′ high frequency energy signal was weakened after the Valsalva maneuver. In addition, we found that the number of effective signals derived from the KS changed in some test results, which may have been directly related to the proficiency and strength of the Valsalva maneuver.

Table 2 shows that when the cardiac ejection volume decreased due to the Valsalva maneuver, the global energy of the KS signal significantly changed. In fact, the mean square error of the low frequency energy ratio decreased by 30.71%, and the same was true for the high frequency energy ratio, which decreased by 23.62%, and the time interval, which decreased by 14.23%. In addition, the mean square error of the total energy ratio increased by 135.53%.

Moreover, the KS extrema also directly varied with cardiac ejection volume. The maximum value of low frequency energy increased by 6.87%, while that of the total energy ratio and high frequency energy ratio decreased by 49.94% and 1.88%, respectively.

A local energy ratio comparison showed that the energy ratio between 50 and 100 Hz, 200–250 Hz, 250–300 Hz, 300–350 Hz, and 350–400 Hz increased by 17.02%, 60.88%, 739.07%, 2647.8%, and 1910.61%, respectively. Conversely, the energy ratio between 100–150 Hz and 150–200 Hz decreased by 59.39% and 52.24%, respectively. Accordingly, it is apparent that the spectral impact of Valsalva maneuver on the KS signal was significantly correlated with frequency, especially as the KS energy increased significantly within the 50–100 Hz and 200 Hz-400 Hz bands. Although the mechanism behind these spectral changes is not clear at present, these phenomena provide a meaningful basis for further research. In addition, the time interval remained unchanged (±2%). This could be explained by the fact that the experiments in this study only involved changes to cardiac ejection and did not have any adverse effects on the volunteers' heart function.

The results of the comparative experiment showed that the Valsalva maneuver had a significant effect on KS. More importantly, a direct correlation between blood flow and KS was demonstrated.

### 4.2. Results of Classiﬁers

The energy features, statistical features, entropy features, and MFCCs features were extracted from KS signal datasets from 115 healthy people and 185 CHF patients. Each KS signal had 48 features in total, which were divided into three datasets: feature set A contained energy features, statistical features, and entropy features; feature set B contained statistical features, entropy features, and MFCCs features; feature set C contained all the features.

We randomly selected 80% of the data as the training set and 20% as the test set. The machine learning algorithms such as TD with fine, medium, and coarse, KNN with fine, medium, and cosine, NB with Gaussian and Kernel, EM with AdaBoost tree, Bagged tree and RUSBoost tree, and the BO-SVM were employed and validated using ten-fold cross-validation on the training set. The performance of each classifier was evaluated on the test set by Acc, Se, Sp, Ps, and F1.

Table 3 shows the performance of each classifier when the feature sets of energy features, statistical features, and entropy features were considered. The coarse DT performed the best among the DT classifiers, with Acc (76.7%), Sp (91.2%), Sp (57.7%), Ps (73.8%), and F1 (90.4%). The second was medium DT, with Acc (75.4%), Se (82.4%), Sp (66.7%), Ps (75.7%), and F1 (83.6%); the fine DT received the lowest score, with Acc (75.0%), Se (82.4%), Sp (65.4%), Ps (75.7%), and F1 (84.4%). The fine KNN has the highest classification accuracy among all the KNN classifiers, with Acc (81.7%), Se (82.4%), Sp (80.8%), Ps (84.8%), and F1 (85.7%); the medium KNN performed secondly, with Acc (78.3%), Se (85.3%), Sp (69.2%), Ps (78.4%), and F1 (86.5%); the cosine KNN came the third, with Acc (76.7%), Se (85.3%), Sp (65.4%), Ps (76.3%), and F1 (86.4%). Among the NB classifiers, the kernel NB performed the best, with Acc (80.0%), Se (82.4%), Sp (76.9%), Ps (82.4%), and F1 (85.2%); the Gaussian NB came the second, with Acc (71.7%), Se (58.8%), Sp (88.5%), Ps (87.0%), and F1 (69.5%). In the EM classifiers, the RUSBoost tree obtained Acc (83.3%), Se (82.4%), Sp (84.6%), Ps (87.5%), and F1 (86.3%); the AdaBoost tree obtained Acc (81.7%), Se (82.4%), Sp (80.8%), Ps (84.8%), and F1 (85.7%); the Bagged tree obtained Acc (80.0%), Se (91.2%), Sp (65.4%), Ps (77.5%), and F1 (90.3%). The performance of BO-SVM was Acc (83.3%), Se (79.4%), Sp (88.5%), Ps (90.0%), and F1 (85.1%).

When statistical features, entropy features, and MFCCs features were taken into consideration, the performance comparison of each classifier is shown in Table 4. When using DT classifiers, the coarse tree had the best performance, with Acc (73.3%), Se (85.3%), Sp (57.7%), Ps (72.5%), and F1 (86.5%), followed by the medium tree, with Acc (71.7%), Se (79.4%), Sp (61.5%), Ps (73.0%), and F1 (82.2%); and the fine tree got Acc (70.0%), Se (76.5%), Sp (61.5%), Ps (72.2%), and F1 (80.0%). Among all KNN classifiers, the medium KNN performed the best, with Acc (78.3%), Se (82.4%), Sp (73.1%), Ps (80.0%), and F1 (84.8%); the fine KNN obtained Acc (73.3%), Se (70.6%), Sp (76.9%), Ps (80.0%), and F1 (76.6%), and the cosine KNN with Acc (73.3%), Se (82.4%), Sp (61.5%), Ps (73.7%), and F1 (84.3%). By using NB classifiers, the best performance was achieved by the kernel NB, with Acc (76.7%), Se (85.3%), Sp (65.4%), Ps (76.3%), and F1 (86.4%), followed by the Gaussian NB, with Acc (75.0%), Se (64.7%), Sp (88.5%), Ps (88.0%), and F1 (74.4%). When the EM classifiers were applied, the RUSBoost tree got the best performance, with Acc (81.7%), Se (88.2%), Sp (73.1%), P (81.1%), and F1 (88.7%); the Bagged tree came the second, with Acc (80.0%), Se (88.2%), Sp (69.2%), Ps (78.9%), and F1 (88.5%), followed by the AdaBoost tree, with Acc (78.3%), Se (85.3%), Sp (69.2%), Ps (78.4%), and F1 (86.5%). The BO-SVM got Acc (80.0%), Se (79.4%), Sp (80.8%), Ps (84.4%), and F1 (83.7%).

Finally, we combined all the features together, including energy features, statistical features, entropy features, and MFCCs features. Each classifier was trained and tested using these features, and the results are displayed in Table 5. Based on the DT classifiers, the best performance was obtained by the fine DT and the medium DT, with Acc (76.7%), Se (73.5%), Sp (80.8%), Ps (83.3%), and F1 (79.4%); coarse DT got Acc (70.0%), Se (67.6%), Sp (73.1%), Ps (76.7%), and F1 (73.7%). The best performance of KNN classifiers was obtained by the cosine KNN, with Acc (83.3%), Se (88.2%), Sp (76.9%), Ps (83.3%), and F1 (89.0%); the fine KNN obtained Acc (80.0%), Se (79.4%), Sp (80.8%), Ps (84.4%), and F1 (83.7%); the medium KNN had the lowest performance, with Acc (78.3%), Se (85.3%), Sp (69.2%), Ps (78.4%), and F1 (86.5%). Using NB classifiers, the Gaussian NB got the performance of Acc (70.0%), Se (67.6%), Sp (73.1%), Ps (76.7%), and F1 (73.7%); and the kernel NB got Acc (76.7%), Se (79.4%), Sp (73.1%), Ps (79.4%), and F1 (82.7%). As the EM classifiers were used, the Bagged tree obtained Acc (83.3%), Se (100%), Sp (61.5%), Ps (77.3%), and F1 (95.7%); the RUSBoost tree obtained Acc (81.7%), Se (76.5%), Sp (88.5%), Ps (89.7%), and F1 (83.1%); and the AdaBoost tree obtained Acc (80.0%), Se (79.4%), Sp (80.8%), Ps (84.4%), and F1 (83.7%). The BO-SVM achieved the best performance of all classifiers, with Acc (85.0%), Se (85.3%), Sp (84.6%), Ps (87.9%), and F1 (88.2%).

Figure 6 depicts the best performance of the five type classifiers across three datasets. The associated classifiers are the fine DT and medium DT on the feature set C, the coarse DT on the feature set A, the cosine KNN on the feature set C, the BO-SVM on the feature set C, Kernel NB on the feature set A, the Bagged tree on the feature set C, and the RUSBoost tree on the feature set A, respectively.

## 5. Discussion

The study on the diagnosis method of heart failure disease based on KS was an early exploratory research. Why were we interested in this? As we know, the KS signal is very easy to collect. Every year, a large number of people take blood pressure tests at home, or in community hospitals and physical examination centers [57]. If these data can be used effectively, it will be of great significance for early noninvasive diagnosis and early warning study of heart failure. It was exciting that the Valsalva maneuver demonstrates a substantial association between cardiac output and Coriolis sound, which gives a solid foundation for our future research, as shown in Table 2 and Figure 5.

In order to achieve the research purpose of this paper, we investigated CHF classification based on multimode KS features. To investigate the influence of different features on classification results, 19 energy features, 12 statistical features, 2 entropy features, and 13 MFCCs features were extracted and divided into three groups. The three sets are as follows: feature set A included 19 energy features, 12 statistical features, and 2 entropy features; feature set B included 12 statistical features, 2 entropy features, and 13 MFCCs features; and feature set C included all features. Five evaluation metrics, that is, accuracy, sensitivity, specificity, accuracy, and F1 score, were used to evaluate each classifier's performance.

Accuracy, sensitivity, and specificity are critical metrics for evaluating medical diagnosis algorithms. Accuracy is the proportion of correctly classified samples to all samples. Sensitivity describes the classifier's ability to identify patients. Specificity indicates the classifier's ability to recognize healthy people [58].

Table 3 shows that the best accuracy when considering the energy feature, statistical feature, and entropy feature was 83.3%, achieved by the BO-SVM classifier and the RUSBoost tree. Both classifiers showed high recognition capabilities for both patients and normal people. Additionally, we can see that there were slight differences between the two classifiers. The sensitivity (82.4%) of the RUSBoost tree was higher than that of BO-SVM (79.4%), while the specificity (84.6%) was slightly lower than that of BO-SVM (88.5%). Fine KNN and AdaBoost tree are the second classifiers, with accuracy, sensitivity, and specificity of 81.7%, 82.4%, and 80.8%, respectively. The RUSBoost tree classifier had the highest classification accuracy of all classifiers, and its sensitivity and specificity were both above 80%. So, in our opinion, the RUSBoost tree outperformed other classifiers in Feature set A.

As we can see in Table 4, when statistical features, entropy features, and MFCCs features were considered, the RUSBoost tree had the highest accuracy of 81.7%, followed by BO-SVM and Bagged tree at 80.0%. The RUSBoost tree and the Bagged tree have higher sensitivity (88.2%) than SVM (79.4%), but their specificity (only 73.1% and 69.2% respectively, less than 80.8% of BO-SVM) is not very excellent. This demonstrates that although the ensemble algorithm was very effective in identifying CHF patients, it had some shortcomings in identifying normal people in Feature set C. Because of its more balanced performance, we believed that BO-SVM outperformed other classifiers in this feature set in terms of accuracy, specificity, and sensitivity.

Results in Table 5 show that, after taking into account all of the energy features, statistical features, entropy features, and MFCCs features, the classifier's accuracy was the highest of all three data sets, at 85.0 %, as achieved by BO-SVM. The second-place classifiers were the Bagged tree and cosine KNN, which had an accuracy of 83.3%. In terms of sensitivity and specificity, BO-SVM had Se (85.3%), Sp (84.6%), Bagged tree had Se (100%), Sp (61.5%), and cosine KNN had Se (88.2%), Sp (76.9%). In Feature set C, BO-SVM also outperformed other classifiers in terms of accuracy, sensitivity, and specificity, offering a high detection rate of CHF and normal people.

According to the results displayed above, BO-SVM performed the best in all three feature sets, with the highest classification accuracy of 85.0% achieved in all the feature sets. Furthermore, we observed that the EM classifiers also performed well in the KS feature classification, frequently outperforming other classifiers. These two algorithms are both excellent classifiers that can be used in KS-based classification.

In terms of the influence of the feature set on classification results, the energy features proposed in this paper had an obvious influence on the classifier's performance. The highest classification accuracy (83.3%) of Feature set A (energy feature, statistical feature, and entropy feature) is higher than that (81.7%) of Feature set B (statistical feature, entropy feature, and MFCCs feature), demonstrating the superiority of energy over MFCCs in KS signal classification. Additionally, the highest classification accuracy of the classifiers reached 85.0% after adding the energy feature to Feature set B (which became Feature set C). As shown in Figure 6, the best performance of all types of classifiers was obtained primarily through Feature set C, demonstrating that the feature data set extraction scheme proposed in this paper is scientifically significant.

Many researchers have made significant achievements in the CHF prediagnosis based on acoustic signals. Although their research object HS differs from the KS of this work, their algorithms and concepts can be used as a reference for this article. As shown in Table 6, CHF classification algorithm based on heart sound had made remarkable achievements, with outstanding classification accuracy, sensitivity, and specificity. Compared with their results, the proposed CHF diagnosis method based on KS signal is not very outstanding in classification accuracy. However, it should be noted that this is the first time we have publicly reported the KS-based CHF diagnosis algorithm, and all of our results are obtained on the clinical measured data set, which makes our findings have clinical guiding significance. As a result, we believe that the proposed method's results in terms of classification accuracy, sensitivity, and specificity are encouraging.

## 6. Conclusions

In this paper, we proposed a CHF prediagnosis method based on the KS signal. Denoising, signal segmentation, and feature extraction methods were established for KS signals, and 19 energy features, 12 statistical features, 2 entropy features, and 13 MFCCs features were extracted. A control experiment was designed to investigate the connection between KS features and CHF disease. Through this experiment, we found that the characteristics of KS changed significantly as cardiac output changed, demonstrating a direct link between the KS signal and CHF disease.

Based on this critical conclusion, we proposed a Bayesian optimization algorithm-based support vector machine model to further investigate the research of CHF classification and compared our method to the conventional machine learning algorithm. A 10-fold cross-validation was used in model training and testing. Each classifier's performance was evaluated using accuracy, sensitivity, specificity, accuracy, and F1 scores. According to our analysis of the performance of each classifier in categorizing the multimodal feature data set, we found that our proposed BO-SVM algorithm performed the best, with Acc (85.0%), Se (85.3%), and Sp (84.6%), followed by Bagged tree, RUSBoost tree, and cosine KNN, with Acc (83.3%), Se (100%), and Sp (61.5%); Acc (83.3%), Se (82.4%), and Sp (84.6%); and Acc (83.3%), Se (88.2%), Sp (76.9%), and Ps (83.3%), respectively. The classifier achieved satisfactory accuracy and met the expected purpose of this paper: early detection of CHF using KS.

These results showed that the early diagnosis algorithm of CHF based on the KS signal proposed in this paper was scientifically significant. In particular, progress toward precise and meaningful KS feature extraction was thoroughly correlated with CHF diagnosis. Although the accuracy is inadequate when compared to the present CHF diagnosis algorithm based on heart sound, we believe that, as a potential analysis approach, our prediction accuracy has room to develop. Moving forward, further machine learning studies should be performed using larger data sets and optimized algorithms. Such studies may enable quick and convenient diagnosis of nondestructive cardiac dysfunction.

## Figures and Tables

**Figure 1:** Classification flowchart for CHF diagnosis based on a KS signal.

**Figure 2:** Flowchart for KS preprocessing.

**Figure 3:** Flow chart of wiener filtering.

**Figure 4:** Schematic diagram of signal location and segmentation results: (a) the denoised KS signal; (b) Shannon envelope of the KS signal; (c) segmentation results from Shannon envelope calculations; (d) segmentation results for the KS signal.

**Figure 5:** Time-frequency comparison of KS before and after the Valsalva maneuver. (a) Original signal. (b) Valsalva signal.

**Figure 6:** The best performance of the models on the three datasets.

**Table 1:** Basic subject information.

Subjects	Ages	SBP	DBP	Num
Healthy	42 ± 22	111 ± 15	73 ± 10	115
CHF patients	61 ± 17	129 ± 35	77 ± 20	185

*Note.* SBP: Systolic Blood Pressure, DBP: Diastolic Blood Pressure, Num: number of the subjects.

**Table 2:** Comparison of KS characteristics before and after the Valsalva maneuver.

KS parameters	Ns	Vm	V(%)
std_enr	12.8	8.89	30.71
std_enr_h	4.99	3.813	23.62
std_TM	19.69	16.89	14.23
std_Ep	7.56	17.81	−135.53
TM_max	104.43	103.25	1.12
TM_min	94.55	96.28	−1.82
enr_max	91.48	97.76	−6.87
enr_min	51.37	69.55	−35.39
enr_h_max	14.05	13.78	1.88
enr_h_min	0.37	0.29	22.70
Ep_max	284.13	142.24	49.94
Ep_min	23.92	23.22	2.921
Stotal(50–100)	75.02	87.79	−17.02
Stotal(100–150)	20.86	8.47	59.39
Stotal(150–200)	3.56	1.70	52.24
Stotal(200–250)	0.46	0.74	−60.88
Stotal(250–300)	0.063	0.53	-739.07
Stotal(300–350)	0.017	0.47	−2647.8
Stotal(350–400)	0.014	0.29	−1910.61

*Note.* Ns: Normal state, Vm: Valsalva maneuver, V: variation.

**Table 3:** Performance of classifiers in feature set A.

Classifier	Acc(%)	Se(%)	Sp(%)	Ps(%)	F1(%)
*DT*					
Fine	75.0	82.4	65.4	75.7	84.4
Medium	75.4	82.4	66.7	75.7	83.6
Coarse	76.7	91.2	57.7	73.8	90.4

*KNN*					
Fine	81.7	82.4	80.8	84.8	85.7
Medium	78.3	85.3	69.2	78.4	86.5
Cosine	76.7	85.3	65.4	76.3	86.4

*NB*					
Gaussian	71.7	58.8	88.5	87.0	69.5
Kernel	80.0	82.4	76.9	82.4	85.2

*EM*					
AdaBoost	81.7	82.4	80.8	84.8	85.7
Bagged	80.0	91.2	65.4	77.5	90.3
RUSBoost	83.3	82.4	84.6	87.5	86.3
BO-SVM	83.3	79.4	88.5	90.0	85.1

**Table 4:** Performance of classifiers in feature set B.

Classifier	Acc(%)	Se(%)	Sp(%)	Ps(%)	F1(%)
*DT*					
Fine	70.0	76.5	61.5	72.2	80.0
Medium	71.7	79.4	61.5	73.0	82.2
Coarse	73.3	85.3	57.7	72.5	86.5

*KNN*					
Fine	73.3	70.6	76.9	80.0	76.6
Medium	78.3	82.4	73.1	80.0	84.8
Cosine	73.3	82.4	61.5	73.7	84.3

*NB*					
Gaussian	75.0	64.7	88.5	88.0	74.4
Kernel	76.7	85.3	65.4	76.3	86.4

*EM*					
AdaBoost	78.3	85.3	69.2	78.4	86.5
Bagged	80.0	88.2	69.2	78.9	88.5
RUSBoost	81.7	88.2	73.1	81.1	88.7
BO-SVM	80.0	79.4	80.8	84.4	83.7

**Table 5:** Performance of classifiers in feature set C.

Classifier	Acc(%)	Se(%)	Sp(%)	Ps(%)	F1(%)
*DT*					
Fine	76.7	73.5	80.8	83.3	79.4
Medium	76.7	73.5	80.8	83.3	79.4
Coarse	70.0	67.6	73.1	76.7	73.7

*KNN*					
Fine	80.0	79.4	80.8	84.4	83.7
Medium	78.3	85.3	69.2	78.4	86.5
Cosine	83.3	88.2	76.9	83.3	89.0

*NB*					
Gaussian	70.0	67.6	73.1	76.7	73.7
Kernel	76.7	79.4	73.1	79.4	82.7

*EM*					
AdaBoost	80.0	79.4	80.8	84.4	83.7
Bagged	83.3	100	61.5	77.3	95.7
RUSBoost	81.7	76.5	88.5	89.7	83.1
BO-SVM	85.0	85.3	84.6	87.9	88.2

**Table 6:** Comparison of CHF classification algorithms based on acoustics.

Authors	Data set	Number of subjects	Method	Performance
Zheng et al.(2015) [59]	Collected by HS acquisition system	88 healthy volunteers and 64 CHF patients	LS-SVM	Acc 95.39%
				Se 96.59%
				Sp 93.75%

Potes et al. (2016) [28]	PhysioNet databases	2575 normal signal and 665 abnormal signal	AdaBoost and CNN	Acc 86.0%
				Se 94.2%
				Sp 77.8%

Gjoreski et al. (2020) [34]	Six (A to F) PhysioNet Challenge datasets & measured HS by digital stethoscope	3153 signals from PhysioNet Challenge datasets &110 healthy people, 51 CHF recorded by digital stethoscope	Machine-learning (ML) and end-to-end Deep Learning(DL)	Acc 92.9%
				Se 82.3%
				Sp 96.2%

Zheng et al. (2022) [35]	Dataset from first Affiliated hospital and the University-Town hospital of Chongqing medical University	51 healthy volunteers and 224 CHF patients	LS-SVM	Acc 82%
				Se 82.1%
				Sp 95.5%

Our method	Dataset of measured KS from the Fourth People's hospital of Zhejiang University	115 healthy subjects and 185 CHF patients	BO-SVM	Acc 85%
				Se 85.3%
				Sp 84.6%

## Data Availability

The data presented in this study are available upon request from the corresponding author. The data are not publicly available due to ethical restrictions.
